# Medical Data Classification Assisted by Machine Learning Strategy

**DOI:** 10.1155/2022/9699612

**Published:** 2022-09-10

**Authors:** Lei Wang, Keqiang Zuo

**Affiliations:** ^1^Zhabei Center Hospital of Jing'an District of Shanghai, Jing'an, Shanghai 200070, China; ^2^The Affiliated Hospital of Jinggangshan University, Ji'an 343000, China; ^3^Shanghai 10th People's Hospital, Tongji University School of Medicine, Shanghai 200072, China

## Abstract

With the development of science and technology, data plays an increasingly important role in our daily life. Therefore, much attention has been paid to the field of data mining. Data classification is the premise of data mining, and how well the data is classified directly affects the performance of subsequent models. In particular, in the medical field, data classification can help accurately determine the location of patients' lesions and reduce the workload of doctors in the treatment process. However, medical data has the characteristics of high noise, strong correlation, and high data dimension, which brings great challenges to the traditional classification model. Therefore, it is very important to design an advanced model to improve the effect of medical data classification. In this context, this paper first introduces the structure and characteristics of the convolutional neural network (CNN) model and then demonstrates its unique advantages in medical data processing, especially in data classification. Secondly, we design a new kind of medical data classification model based on the CNN model. Finally, the simulation results show that the proposed method achieves higher classification accuracy with faster model convergence speed and the lower training error when compared with conventional machine leaning methods, which has demonstrated the effectiveness of the new method in respect to medical data classification.

## 1. Introduction

Disease diagnostic analysis is a highly specialized and time-consuming task, which is prone to inconsistencies between and within observers [1, 2]. Computer-aided diagnosis can reproduce the diagnostic process and reduce the subjectivity of observers to improve the reliability of results. Medical data classification is used to solve problems related to disease. The main goal is to extract clinically relevant pathological information or knowledge from medical data. Nowadays, with the development of technology, the huge amount of medical data generated by clinical practice makes data-driven high-precision computer-aided diagnosis possible [3].

How to mine valuable information from increasingly abundant data has become a research hotspot in the field of artificial intelligence. Data mining (DM) is one of the most powerful data analysis methods at present. Through DM, it can extract the hidden but unknown and potentially useful information from data to discover rules or patterns [4]. In recent years, various DM techniques have been widely used in data analysis tasks. DM technology has been applied to medical data research since it was proposed. As the object of medical research gradually changes from clinical diagnostic data to bioinformatics data, medical data mining has increasingly become one of the most active research and application fields [5]. Clinical diagnostic data contain a large amount of valuable information. Data mining of clinical diagnostic data of patients with different diseases is helpful to discover the risk factors related to the disease and their interaction, which can provide reference for clinical diagnosis and treatment of the diseases [6].

With the increasing progress of science and technology, people now rely more and more on computers to obtain all kinds of information and use computer technology to solve all kinds of classification problems encountered. In recent years, numerous statistical methods and disease risk factor analysis, including principal component analysis (PCA), logistic regression, linear discriminant analysis (LDA) and support vector machine (SVM), and many innovative research results have been obtained [7, 8]. However, since clinical data has the characteristics of high dimensional feature space, high redundancy, and strong correlation between data features, many classical classification algorithms are not ideal for the classification accuracy of medical datasets.

In recent years, deep learning models have made breakthroughs in data mining, artificial intelligence, data classification, and other fields. The deep learning model is generally a deep neural network composed of multiple processing layers, which can learn data representation and data features with multiple layers of abstraction [9]. Traditional machine learning classification methods are based on shallow structure algorithms, which cannot express complex function features in the case of limited data samples, and there is a problem of low model generalization ability in complex data classification [10, 11]. Deep neural network model can represent the deep nonlinear network structure and further approximate complex functions. It has the ability to learn the essential characteristics of data samples from a small number of data samples. The basic neural network model consists of many units that are simply interconnected called neurons, and a single neuron generates a single real-valued activation sequence [12]. Deep neural network generally adopts the gradient descent method to guide the updating of network parameters, which is used to represent the features obtained by the current layer from the previous layer and then passed down to the next layer. The neural parameters of each layer of the network model only affect the parameters of the next layer of the network model. The output results of the output layer are compared with the label, and the training error can be minimized by adjusting the connection weights of neurons in each layer of the network model [13, 14]. In practical applications, as most of the multilayer structures contain multiple nonlinear processing units, it often leads to the local minimum solution of the nonconvex cost objective function, and the final classification accuracy is lower than that of other machine learning algorithms. In view of this common problem, many new deep neural network models have been proposed through further research [15, 16].

In current studies, representative ones are recurrent neural network (RNN), long- and short-term memory (LSTM), CNN, restricted Boltzmann machine (RBM), etc., among which CNN is one of the most widely used deep learning models in recent years [17, 18]. Its main feature is that in the network model, the two layers are fully connected, and there is no connection within the layer. CNN is quite popular due to its excellent data feature extraction ability. Aiming at the complex characteristics of medical data and the advantages of CNN, this paper mainly studies the medical data classification algorithm based on the CNN model. While maintaining or improving the classification performance of the classification algorithm, the running time of the algorithm is reduced, so that the data mining results have better transparency and understandability [19, 20]. This research belongs to the interdisciplinary research of computer science and biological information. The research results can not only enrich machine learning and data mining algorithms but also promote the application of data mining and machine learning technology in the medical field and provides scientific basis and decision support for medical experts to determine treatment plan and carry out medical research. The reminder of this paper is as follows: Section 2 gives the related work, and Section 3 is the machine learning-based medical data classification algorithm. And the experimental results and analysis are given in Section 4. Finally, Section 5 concludes the paper.

## 2. Related Work

Two important research directions of medical data mining are clinical data mining and biological information data mining. For clinical diagnostic datasets, data mining mainly uses feature selection and machine learning algorithms to explore disease risk factors, which affects the occurrence of certain diseases and provides decision support for doctors to make clinical diagnosis and reasonable treatment plans [21].

### 2.1. Shallow Neural Network Classifier

Machine learning has been widely used to analyze biomedical data and classification tasks [22, 23]. Classification is an important problem in supervised learning in machine learning. For nonlinear classification, the inner product between instances can be changed into kernel function, so that the problem can be transformed into a linear classification problem in a specific dimensional feature space, so that linear support vector machines can be learned in a high dimensional feature space. SVM has been widely used in neuroscience and bioinformatics because the algorithm can process high-dimensional data. The main disadvantage of this method is that it is easy to overfit due to the large amount of calculation. Logistic regression aims at a combination of variables to maximize the probability of predicting the expected outcome [24]. Maximum likelihood estimation is used for parameter estimation, and likelihood ratio test is used for significance test. In order to avoid overfitting and improve generalization ability, logistic regression and regularization are often used in combination by adding a penalty term to optimize the objective function, reducing the size of parameters corresponding to features. Logistic regression can get approximate probability prediction in addition to categories, which has the advantages of simple, efficient, easy to interpret, and easy to expand, and is widely used in the classification tasks of bioinformatics.

The random forest algorithm is based on the idea of ensemble learning to integrate multiple trees. Its basic unit is decision tree. For classification problems, each decision tree is a classifier that learns and makes predictions independently. The random forest algorithm integrates the results of all classification and then begins to vote to further obtain more accurate classification. The predicted variance is inversely proportional to the number of independent trees in it. Random forest classifier has been widely used in bioinformatics [25]. One of its main advantages is that it can evaluate the importance of each feature in classification while determining categories. One of its disadvantages is its sensitivity to input parameters. Naive Bayes is a probability classifier based on Bayes theorem, which adopts the assumption of attribute condition independence. Naive Bayes builds conditional probabilities of features under each class and determines the most likely categories for features of test data. The advantage of naive Bayes is that it still has a fast running speed in the face of a large amount of training and test data. However, when the assumption is not met, there is no guarantee that it will perform well. This algorithm has many applications in bioinformatics. Multilayer perceptrons, also known as artificial neural networks (ANN), map multiple datasets of inputs to a single dataset of outputs [4]. Neurons make up an artificial neural network, each layer of which is connected by weight, also known as a synapse. The advantage of multilayer perceptron is that the number of neurons and hidden layers can be designed according to the complexity of the target dataset. Generally, the more complex the target dataset, the more hidden layers are needed for feature extraction. However, in the multilayer perceptron, the layers are fully connected, which makes it difficult to update parameters.

### 2.2. Deep Neural Network Classifier

Deep learning refers to the machine learning process in which a multilevel network structure representing the characteristics of the data is obtained by applying some specific training methods to the data samples. Deep learning network structure of the model is composed of a large number of neurons connected to each other, measured by weight connection strength between neurons connected to each other. Through the change of weight value in the process of model training so as to achieve the aim of function of the control model, the sizes of the neurons in essence are all in the neural network model which is for calculating the required minimum unit [26]. In recent years, deep learning methods have attracted extensive attention in the fields of pattern recognition and machine learning. The deep neural network model is a computing model composed of multiple processing layers, which extracts effective learning features from data [27]. As an important tool of artificial intelligence, the deep learning model has shown great potential. The theory and application of deep learning have attracted extensive attention in the international and domestic academic circles, and many famous enterprises in the world also attach great importance to the research and application of this aspect. For example, Tesla withdrew from self-driving cars based on deep learning, and Baidu, a Chinese Internet giant, set up a deep learning research institute to implement the technological research results of artificial intelligence.

Large-scale natural datasets have greatly promoted the development of deep learning technology. Deep learning can be used to complete the classification of medical image data [28]. However, its development is limited by data. The scale of medical image data is often limited. When there is enough data, all parameters in the neural network can be randomly initialized and then trained. Another strategy is transfer learning. Another strategy is transfer learning, which fine-tunes the parameters of the network model trained in advance on external datasets. Most studies using transfer learning strategies replace and retrain the deepest layer of the network, while the shallow layer is a variation of the transfer learning strategy fixed after the initial training, which combines fine-tuning and deep feature methods. Fine-tune the pretrained network on new datasets to obtain deeper features [29]. Deep neural networks (DNN) re a discriminant model, which can be trained with the backpropagation algorithm, and weight updating can be solved by stochastic gradient descent. In a broad sense, DNN is the general term of deep learning, including a series of other neural network structures, such as convolutional neural network and recurrent neural network. Chivalrous DNN refers to a network structure with only full connections. Based on the above discussions, the main contributions of this work can be concluded as below:

1. The method in this paper is based on the depth model and can deal with the classification of large-scale medical data
2. Experimental results show the effectiveness and practicability of the proposed method. That is to say, the method in this paper has both theoretical and practical significance

## 3. The Machine Learning-Based Medical Data Classification Algorithm

The earliest feedforward neural network is also called multilayer perceptron (MLP), which is the simplest neural network model and given in Figure 1. From the figure, we know that the MLP contains the input layer, hidden layer, and output layer. And each neuron is arranged in layers. As the simplest neural network at that time, each neuron is connected to the upper layer,the output of the upper layer continues as the input of the lower layer, and there is no feedback between layers.

The MLP neural network is given in here, from which we can see that neural network can be divided into three parts: input layer, hidden layer, and output layer according to its different functions. Due to the shallow network layer and the use of linear activation units, the early fully connected neural network models are often unable to solve complex problems.

### 3.1. Deep CNN Model for Medical Data Classification

Based on the traditional full-connection layer neural network, CNN adds convolution layer and pooling layer to form the deep CNN model, which is shown in Figure 2.

The function of the convolution layer lies in the extraction of image features. The essence of the convolution kernel is a filter matrix, which can produce many different effects on the original image. The calculation process of convolution is shown below:

(1) $$\begin{array}{c} {\text{CONV}}_{\left(ij\right)}=\overset{m-1}{\underset{i}{\sum }}\overset{n-1}{\underset{j}{\sum }}u_{ij}\times w+b\;\left(i=1,2\cdots m-1;j=1,2\cdots n-1\right), \end{array}$$

where *u*_*ij*_ is the input image, *m* and *n* are the size of the input image, *w* is the size of the convolution kernel, and *b* is the bias constant of the convolution kernel. CONV (*ij*) is the characteristic graph output after convolution operation.

CNN adds an activation function layer to the network and analyzes the model better by adopting the feature mapping method of nonlinear function.

(2) $$\begin{array}{c} f\left(x\right)=\frac{1}{1+e^{-x}}. \end{array}$$

The mathematical expression of tanh function is

(3) $$\begin{array}{c} f\left(x\right)=\frac{e^{x}-e^{-x}}{e^{x}+e^{-x}}. \end{array}$$

The mathematical expression of ReLU function is

(4) $$\begin{array}{c} f\left(x\right)=\max\left(0,x\right). \end{array}$$

The full name of ReLU function is rectified linear unit. The function is one of the commonly used activation functions, which is characterized by low computational complexity and no exponential operation. However, it is worth noting that although ReLU function has certain advantages, it also has some shortcomings in the actual calculation process. When the data passes through the negative range of ReLU function, the output value is equal to 0. The Leaky-ReLU function can solve the above problem.

(5) $$\begin{array}{c} f\left(x\right)=\left\{\begin{array}{cc} x, & x\geq 0,\\ \alpha x, & x<0. \end{array}\right. \end{array}$$

Therefore, the efficiency of the entire network operation can be improved to a certain extent. The corresponding equations of *sig* and *tanh* are as follows:

(6) $$\begin{array}{c} \left\{\begin{array}{c} sig\left(x\right)=\frac{1}{1+\exp\left(-x\right)},\\ \tanh\left(x\right)=\frac{\exp\left(x\right)-\exp\left(-x\right)}{\exp\left(x\right)+\exp\left(-x\right)}, \end{array}\right. \end{array}$$

(7) $$\begin{array}{c} h_{w,b}\left(x_{i}\right)=\left[\begin{array}{c} p\left(y_{i}=1\left|x_{i};w,b\right.\right)\\ p\left(y_{i}=2\left|x_{i};w,b\right.\right)\\ p\left(y_{i}=3\left|x_{i};w,b\right.\right)\\ \cdots \\ p\left(y_{i}=n\left|x_{i};w,b\right.\right) \end{array}\right]=\frac{1}{\sum_{j=1}^{n}e^{w_{j}x_{i}+b_{j}}}\left[\begin{array}{c} e^{w_{1}x_{i}+b_{1}}\\ e^{w_{2}x_{i}+b_{2}}\\ e^{w_{3}x_{i}+b_{3}}\\ \cdots \\ e^{w_{n}x_{i}+b_{n}} \end{array}\right]. \end{array}$$

The output layer adopts softmax function to normalize, and the probability value *h*_*w*,*b*_(*x*_*i*_) in the corresponding category is shown in (7). In classification tasks, it is a common method to use crossentropy loss function to evaluate the gap between predicted value and true value. The crossentropy (CE) formula is as follows:

(8) $$\begin{array}{c} \text{loss}=-\frac{1}{m}\overset{m}{\underset{j=1}{\sum }}\overset{n}{\underset{i=1}{\sum }}y_{ji}\log\left({\hat{y}}_{ji}\right). \end{array}$$

The error calculated from the CE function needs to be calculated by back propagation, so as to realize the newer back propagation of model parameters. The original form of the gradient descent method is shown below:

(9) $$\begin{array}{c} \theta ≔\theta -\alpha \frac{\partial }{\partial \theta }J\left(\theta \right), \end{array}$$

where the *θ* is a parameter. In the experiments in the following chapters, this paper also verifies that the use of Adam has faster convergence than SGD. The mathematical expression of a common Adam optimizer is given as

(10) $$\begin{array}{c} m_{t}=\beta_{1}m_{t-1}+\left(1-\beta_{1}\right)g_{t},\\ v_{t}=\beta_{2}v_{t-1}+\left(1-\beta_{2}\right)g_{t}^{2}. \end{array}$$

And the *β*_1_ and *β*_2_ are all parameters, and *m*_*t*_ and *v*_*t*_ are the wanted value. Therefore, the updating rule of gradient descent is as follows:

(11) $$\begin{array}{c} \theta_{t+1}=\theta_{t}-\frac{\alpha }{\sqrt{v_{t}+\epsilon }}m_{t}. \end{array}$$

Based on the above discussions, the proposed medical data classification algorithm in this work is shown in Figure 3. It mainly includes data preprocessing, CNN model establishment, judgment of stop conditions, and final classification results.

## 4. Experimental Results and Analysis

### 4.1. Experimental Data Introduction

To verify the effectiveness of the proposed algorithm, three representative medical datasets were selected from the UCI dataset, which have been widely cited in the literature [29]. Among them, breast dataset is a breast cancer dataset from clinical cases, including 699 samples, 9 numerical variables, and 1 classification variable. The target variable is the category of samples: benign and malignant. Liver is a very different dataset with 395 samples, including 6 numerical variables and 1 target variable. Diabetes is a diabetes dataset, which is a constrained selection dataset consisting of 768 samples of descendants of Pima Indians older than 21 years, each containing 8 numerical variables and 1 categorical variable.

In addition, in order to better compare the test results, all the data were preprocessed, including noise removal, anomaly removal, and normalization processing, so as to obtain pure and directly usable data, which helped to improve the classification performance of the subsequent model.

### 4.2. Experimental Result Analysis

In order to demonstrate the universality of the proposed method, change curves of different activation functions of the CNN model are presented in Figure 4. As can be point out from the figure, under the dataset of this paper, different activation functions have different characteristics, but they all have the following common characteristics: (1) differentiability: this property is a prerequisite when using gradient-based optimization algorithms to optimize models and (2) monotonicity: when the activation function meets the monotonicity, the single-layer network is guaranteed to be convex, so that the subsequent convex optimization operations can be carried out. But in this case, the learning rate usually needs to be set to a small value, which inevitably increases the training time. Based on the above, the ReLU function is selected in this paper.

Apart from training errors, Figure 5 shows the effects of network layers on test accuracy and model testing time, the left is the effects on testing accuracy, and the right is the effects on model testing time: (a) test accuracy and (b) testing time. From the figure we know that with the increase of network layers, both test accuracy and test time show a normal distribution trend. In particular, when the number of network layers is 20, the test accuracy of the model reaches the highest, about 90%, while when the network layers is 100, the test accuracy reaches the lowest 18%. Similarly, when the number of network layers is 20, the test time of the model is the fastest 2.5 minutes. With the increase of the number of layers, the test time of the model becomes longer and longer. When the number of layers is 100, the test time of the model is the longest 9.3 minutes. From the above analysis, it can be seen that the selection of appropriate network structure is important.

Base on the above model setting, the classification results of three kinds of medical data by different methods are drawn as shown in Figure 6. Similarly, samples 1-400, 401-800, and 801-1200 on the abscissa are disease 1, disease 2, and disease 3, respectively, and the ordinate represents labels for medical data. From the figure, we know that the classification accuracy of the proposed CNN model method for disease data 1, 2, and 3 is 97.5%, 99.5%, and 92.25%, respectively. In addition, the average classification accuracy of CNN is much better than that of the SVM algorithm (96.42% compared with 65.92%, 68.83%, 76%), which also proves the effectiveness of the proposed method from another perspective.

To further demonstrate the classification performance of the CNN approach, the relationship between model complexity and iteration times is given in Figure 7. Among them, the model has the fastest increase in memory requirements; so, the method proposed in this paper is based on the deep learning model, which has higher requirements on hardware computing capacity but can achieve better model performance. However, time complexity, space complexity, and computational efficiency all show a slow growth trend, which shows the practicality and reliability of the method presented in this paper.

Finally, Figure 8 shows the relationship between classification accuracy and iteration times of different methods. We can see from the figure that with the increase of iteration number, the classification performance of the three methods shows an increasing trend. When the iteration number is 600, the three models all reach the highest classification accuracy, which is 79%, 88,% and 97%, respectively. Therefore, the CNN model in this paper achieves the highest classification accuracy. In addition, even when the number of iterations is small, the proposed method also has the best model performance and achieves the highest classification accuracy throughout the training process, which demonstrates the effectiveness of the proposed method in medical data classification.

## 5. Conclusions

Data classification plays an important role in medical data processing and has been applied in many fields. Medical data classification problems are diverse and complex and are easily affected by noise and instrument defects in the process of data analysis, which will greatly affect the doctor's judgment of the lesion location. Therefore, how to improve the effect of medical data classification is conducive to the development of technology and practical application.

This paper introduces the background information of medical data classification and the development trend of classification technology at the present stage and introduces the relevant knowledge points. On this basis, the medical data classification method based on the CNN model is proposed in this paper, and the classification effect is good. Specifically, the method proposed in this paper achieved the best classification accuracy (97.5% 99.5%, and 92.25% for disease data 1, 2, and 3, respectively) and fastest running speed. In addition, it can be seen that the parameters of the CNN algorithm are relatively high; so, the next step will focus on improving the operation effect of the CNN algorithm while reducing parameters. And other physiological data about the patient can also be taken into account.

## Figures and Tables

**Figure 1:** The conventional multilayer perceptron network.

**Figure 2:** The typical schematic diagram of CNN neural network.

**Figure 3:** The overall process of the proposed method.

**Figure 4:** Different activation functions curves of the CNN model.

**Figure 5:** The influence of network layers on test accuracy and model testing time: (a) test accuracy and (b) testing time.

**Figure 6:** Classification results of the three kinds of disease by the CNN model.

**Figure 7:** The relationship between model complexity and iteration times.

**Figure 8:** The relationship between classification accuracy and iteration times of different methods.

## Data Availability

The experimental data used to support the findings of this study are available from the corresponding author upon request.
